This article has been retracted.

# A Retrospective Study on the Time in Range of Blood Glucose and Type 2 Diabetic Peripheral Neuropathy

**DOI:** 10.1155/2022/2743679

**Published:** 2022-07-28

**Authors:** Ming Li, Kaiming Wu, Jianfei Chang, Wan-chen Jiang

**Affiliations:** ^1^Endocrine Department, First Affiliated Hospital, Heilongjiang University of Chinese Medicine, Harbin 150000, China; ^2^Isotope Department, First Affiliated Hospital, Heilongjiang University of Chinese Medicine, Harbin 150000, China; ^3^Endocrine Department, The Third Affiliated Hospital of Heilongjiang University of Chinese Medicine, Harbin 150000, China; ^4^Heilongjiang University of Chinese Medicine, Harbin 150000, China

## Abstract

**Background:**

Time in range (TIR) is one of the basic indicators to assess glycemic control. In this study, the TIR of DPN patients was used as the observation index to further evaluate the correlation between TIR and DPN, so as to provide new ideas for preventing the occurrence of DPN and delaying its disease progression.

**Methods:**

A total of 120 patients with T2DM (T2DM) who were hospitalized in the Endocrinology Department of our hospital from October 2018 to February 2020 were included and divided into two groups according to whether the nerve conduction velocity was normal or not, the diabetic peripheral neuropathy group (DPN) and the other groups. No diabetic peripheral neuropathy group (NDPN). According to the corresponding inclusion and exclusion criteria, the baseline data were recorded, and test indicators such as homocysteine and blood lipids were collected at the same time, and TIR was collected by a transient blood glucose meter. To explore the relationship between TIR and other indicators and peripheral neuropathy in T2DM.

**Results:**

A total of 120 T2DM patients participated in the study, including 82 in the DPN group and 38 in the NDPN group. There were no statistically significant differences in basic indicators such as age, height, and weight between the two groups. Glycated hemoglobin (HbA1c) and homocysteine (Hcy) in DPN group were higher than those in NDPN group, while TIR and HDL-C were lower than those in NDPN group (*P* < 0.05). Logistic regression analysis showed that HbA1c and Hcy were risk factors for DPN, and TIR and HDL-C were protective factors for DPN, with statistical significance (*P* < 0.05). The prediction results of TIR, Hcy, HDL-C, and HbA1c on diabetic peripheral neuropathy were analyzed by ROC curve, and the prediction results of the five variables were all statistically significant (*P* < 0.05) and have a better prediction effect.

**Conclusion:**

(1) The results of TIR level suggest that the longer the blood sugar is in the good control range, the more beneficial it is to reduce the occurrence of DPN. (2) TIR and HDL-C are protective factors for DPN, and HbA1c and Hcy are risk factors for DPN. (3) The results of ROC curve analysis showed that TIR, Hcy, HbA1c, and HDL-C had a good predictive effect on the occurrence of DPN.

## 1. Introduction

According to the World Health Organization, the number of people with diabetes worldwide will reach 360 million by 2030, and diabetes-related complications also seriously affect the quality of life of patients [1, 2]. Therefore, finding an effective measure of DPN can prevent the development of this complication [3, 4]. TIR is an indicator for evaluating blood sugar control. The longer the TIR time, the better the blood sugar control [5, 6]. Glycated hemoglobin has always been the golden indicator to reflect blood sugar control [7]. However, due to the interference of many conditions such as anemia and pregnancy, it cannot reflect the rapid changes in blood sugar in a short period of time [8, 9]. The TIR is not interfered by the average blood sugar level and other pathological factors and can describe the blood sugar control level more realistically [10]. The scanning glucose monitoring system is a new type of blood glucose monitoring mode after glycosylated hemoglobin and self-monitoring of blood glucose (SMBG).

In this study, by observing the basic clinical data of patients with T2DM (T2DM), the related risk factors and protective factors of DPN, the correlation between serum TIR and DPN, and the effective indicators for predicting the occurrence of DPN were investigated.

## 2. Materials and Methods

### 2.1. Diagnostic Criteria

The diagnostic criteria for T2DM adopts the T2DM diagnostic criteria issued by the World Health Organization (WHO) in 1999 [11]. Among them, the diagnostic criteria of DPN: mainly exclusion diagnosis. Since polyneuropathy is the most common type of diabetic peripheral neuropathy, this study adopted the American Diabetes Association's 2017 “position statement” for diabetic neuropathy [12]. After summarizing, it is adopted: patients with diabetes who have typical symptoms or signs of peripheral neuropathy (feelings such as burning sensation in distal limbs, abnormal pain and temperature, pressure, vibration and ankle reflexes, and are symmetrical) can be in clinical diagnosis. In the absence of typical clinical manifestations, neuroelectrophysiological examination is used. When there is abnormal nerve conduction function, other diseases that can lead to neuropathy should be excluded systemic diseases such as vascular disease, metabolic system diseases caused by metabolites affecting neuropathy such as increased creatinine, inflammatory lesions such as chronic inflammatory demyelinating disease, nutritional lesions, and infectious lesions after diagnosis.

Definition of hyperhomocysteinemia (HHcy) [13]: blood homocysteine > 15 *μ*mmol/L was defined as HHcy; otherwise, it was nonhomocysteine (NHHcy).

Definition of blood glucose time in target range (TIR) [14]: refers to the time that blood sugar is within the target range (usually 3.9 to 10.0 mmol/L). The upper limit of TIR is set in line with the internationally recommended postprandial blood glucose standard value for diabetic patients, and the lower limit reflects the diagnostic value of hypoglycemia in diabetic patients.

### 2.2. Inclusion of the Exclusion Criteria

Inclusion criteria for this study: (1) age ≥ 18 years; (2) meet the diagnostic criteria for T2DMDPN.

Exclusion criteria for this study: (1) patients with severe systemic diseases such as tumors and severe infections; (3) acute complications of diabetes such as diabetic ketoacidosis; (4) patients with abnormal thyroid function; (5) taking folic acid, vitamin B_12_, methotrexate, and other drugs that affect peripheral nerves; (6) sequelae of cerebrovascular disease, lumbar vertebral disease, etc.; (7) peripheral neuropathy caused by long-term heavy drinking; (8) patients who cannot cooperate.

### 2.3. General Patient Data

The research subjects were selected from T2DM patients who were hospitalized in the Endocrinology Department of our hospital from October 2018 to February 2020. The screening process is shown in Figure 1. Each included subject signed an informed consent form, which was reviewed and approved by the Ethics Committee of our hospital. There were no statistically significant differences in basic indicators such as age, height, and weight between the two groups. After screening for inclusion and exclusion criteria, a total of 120 T2DM patients were included in this study, of which 82 were included in the DPN group and 38 cases in the NDPN group; the general data of the two groups are shown in Table 1.

### 2.4. Observing Indicators

Blood samples were collected overnight on an empty stomach: high-density lipoprotein cholesterol (HDL-C), triglyceride (TG), total cholesterol (TC), low-density lipoprotein cholesterol (LDL-C), homocysteine (Hcy), etc.; the above indicators should be detected by an automatic biochemical analyzer. Glycated hemoglobin (HbA1c) was determined by electrochemiluminescence. Patients' TIR levels were acquired using the Abbott FreeStyleLibreH scanner and probe. Nerve potentials were induced by Keypoint 4-channel nerve potential meter. The motor nerve detection included the ulnar, median, tibial, and common peroneal nerves, and the sensory nerve detection included the ulnar, median, common peroneal, and superficial peroneal nerves. We followed up all patients for 3 months after this.

### 2.5. Statistical Methods

The research data were analyzed using SPSS 22.0 statistical software. When the measurement data are continuous data, and meet the normal distribution and homogeneity of variance, the data is expressed in the form of (*x* ± SD), and the analysis uses two independent samples Student's *t* test; when the measurement data is nonnormal distribution, the medium numerical and interquartile range method M (P25, P75) description, using Mann–Whitney *U* test; enumeration data expressed as percentage, using chi-square test; binary logistic regression was used to analyze DPN risk factors and protective factors; using GraphPad Prism8 made a forest plot model of the credible interval of binary logistic regression; and applied ROC curve to analyze the specificity and sensitivity of the influencing factors of DPN. The test results were considered statistically significant at *P* < 0.05.

## 3. Results

### 3.1. Correlation between Different TIR Levels and the Incidence of DPN

According to the level of TIR, they were divided into T1 group: HbA1c ≤ 6.0 h/d, T2 group: HbA1c > 6.0 h/d, and the incidence of DPN was about 39% and 79%, respectively. Correlation analysis was used to explore the correlation between TIR levels and the incidence of DPN. It was found that there was a significant correlation between TIR and DPN, with a correlation coefficient of 0.471, and a positive correlation, significant *P* < 0.01 (see Figure 2 and Table 2).

### 3.2. Correlation between Different Hcy Expression Levels and the Incidence of DPN

The patients were divided into two groups according to the blood Hcy level, namely, the HHcy group and the NHHcy group. The incidence of DPN in the two groups was about 98.5% and 36.2%, respectively. Correlation analysis was used to explore the correlation between Hcy levels and the incidence of DPN. It was found that there was a significant correlation between Hcy and DPN, with a correlation coefficient of 0.60, and a positive correlation, significant *P* < 0.01 (see Figure 3 and Table 2).

### 3.3. Analysis of Influencing Factors of DPN

Binary logistic regression analysis of factors affecting DPN showed that HbA1c and Hcy were risk factors for DPN, while TIR and HDL-C were protective factors for DPN, with statistical significance (*P* < 0.05) (see Table 3). Other variables were not statistically significant (*P* > 0.05).

### 3.4. ROC Curve Analysis of the Influencing Factors of DPN □□

By using the ROC curve, the prediction results of TIR, Hcy, HDL-C, and HbA1c for diabetic retinopathy were analyzed, and the prediction results of the four variables were all statistically significant (*P* < 0.05). All have good predictive effects; their respective sensitivities and specificities are expressed by coordinates as (0.61, 0.97), (0.90, 1.00), (0.82, 0.94), and (0.73, 0.74), and the critical values are expressed as 68.50, 9.35, 8.35, and 6.75; at this critical value point, each index predicts the best effect of DPN (see Figure 4 and Table 4).

## 4. Discussion

DPN is one of the most common chronic complications of diabetes [15, 16]. It is characterized by insidiousness and difficulty to detect. About 50% of T2DM patients are affected, and the disease is irreversible at the time of discovery [17, 18]. Some studies have shown that blood glucose fluctuation is an independent risk factor for chronic complications in T2DM patients and promotes the occurrence of DPN through mechanisms such as oxidative stress and endothelial damage [19, 20]. The 120 patients included in this study were divided into DPN group and NDPN group according to the inclusion criteria, and the baseline data and research indicators of the two groups were compared. In the DPN group, the levels of HbA1c and Hcy were higher than those in the NDPN group, while the levels of TIR and HDL-C were lower than those in the NDPN group, and the difference was statistically significant. Logistic regression analysis was used to observe the effects of Hcy, BMI, TIR, diabetes duration, and other indicators on DPN. After adding the above indicators into the equation, the results showed that HbA1c and Hcy were risk factors for type 2 diabetic peripheral neuropathy and TIR and HDL-C A protective factor for diabetic peripheral neuropathy.

The results of this study used correlation analysis to explore the correlation between TIR levels and the incidence of DPN. It was found that there was a significant correlation between TIR and DPN. The ROC curve was used to analyze the effects of TIR, Hcy, HDL-C, and HbA1c on diabetic retinopathy. The prediction results showed that the prediction results of the four variables were all statistically significant. The above results suggest that TIR has a protective effect on the complications of T2DM patients, and may coordinate with factors such as Hcy, HDL-C, and HbA1c to regulate the blood glucose homeostasis of patients. Previous studies have shown that, compared with glycated hemoglobin, TIR can not only reflect blood sugar fluctuations, hyperglycemia, hypoglycemia, and other dimensions of blood sugar control but also is not interfered by physiological or pathological factors such as anemia and pregnancy and is more accurate and efficient [21, 22]. A survey of 3,461 people with diabetes showed that TIR was second only to food among the factors that participants felt had a major impact on their daily lives [23]. This study provides a basis for enhancing patient compliance and controlling blood sugar to the target. These studies complement the results of this experiment.

Study shows that hyperhomocysteinemia is significantly associated with macrovascular complications in diabetic patients [24, 25]. However, whether the reduced homocysteine level can reduce the occurrence of DPN is rarely mentioned in previous literature studies. This experimental study shows that with the increase of Hcy level, the prevalence of DPN gradually increases, and plasma Hcy is related to abnormal nerve conduction velocity. This is consistent with previous studies [26, 27]. When Hcy > 15 *μ*mmo/L, the nerve conduction velocity obviously decreases with the increase of Hcy, and there is a significant correlation between the two [21, 28]. This may be related to high Hcy leading to oxidative stress, endothelial cell damage, and neurotoxicity damage. In addition, it may also be related to insulin deficiency and resistance affecting protein metabolism. Insulin promotes protein synthesis [29, 30]. In the absence of insulin, the conversion of Hcy to its precursor amino acid is reduced [31, 32]. The decrease in insulin level in DPN patients leads to the increase of Hcy [33, 34]. Whether early intervention to reduce Hcy levels in NDPN can delay the progression of DPN remains to be studied. Due to the small sample size of this study, the correlation analysis between Hcy levels and TIR was not performed.

In conclusion, TIR is a protective factor for type 2 diabetic peripheral neuropathy, and Hcy and HbA1c are risk factors for DPN. At the same time, the levels of Hcy and HbA1c in DPN patients were significantly higher than those in the control group, and there was a significant correlation between HbA1c and DPN. TIR, Hcy, HbA1c, and HDL-C have good predictive effect on the occurrence of type 2 diabetic peripheral neuropathy.

## 5. Limitations

There are some imperfections in this study, including a small sample size, few data, and a cross-sectional controlled study, which cannot determine the causal relationship, and the results may be biased. Conduct: this study did not compare the blood sugar fluctuations and the improvement of neuropathy symptoms in the patients who were given supplements such as folic acid and vitamin B_12_, and further research is needed.

## 6. Conclusion

1. The results of TIR level suggest that the longer the blood sugar is in the well-controlled range, the more beneficial it is to reduce the occurrence of DPN
2. TIR and HDL-C are protective factors for DPN, and HbA1c and Hcy are risk factors for DPN
3. The results of ROC curve analysis showed that TIR, Hcy, HbA1c, and HDL-C had a good predictive effect on the occurrence of DPN

## Figures and Tables

**Figure 1:** Experiment participant screening process.

**Figure 2:** Incidence of DPN in T1 and T2 groups. ^∗^*P* < 0.05, compared with NHHcy group (unit of NHHcy and HHcy: mmol/L).

**Figure 3:** Incidence of DPN in HHcy and NHHcy groups.

**Figure 4:** The ROC curves of the factors affecting the DPN.

**Table 1:** General information of patients (*x* ± *s*).

Characteristics	DPN group (*n* = 82)	NDPN group (*n* = 38)
Gender (male/female)	42/40	18/20
Age (age)	58.7 ± 6.6	60.3 ± 7.0
Stature (cm)	165 ± 10.7	168 ± 12.5
BMI	26.09 ± 1.3	25.24 ± 2.1
Disease course (month)	8.7 ± 4.6	10.1 ± 3.5
Fasting blood glucose (mmol/L)	8.7 ± 1.1	9.1 ± 1.3
Blood glucose after 2 h (mmol/L)	12.5 ± 2.0	12.8 ± 1.8

**Table 2:** Association analysis between DPN incidence and HbA1c levels and Hcy levels.

Dependent variables	Independent variables	*R*	*P*
DPN	TIR	0.47	<0.01
	Hcy	0.60	<0.01

**Table 3:** Regression analysis of the factors affecting the DPN.

	*β*	OR	95% CI	*P*
HbA1c	1.47	4.62	(1.77, 10.18)	0.02
HDL-C	-4.43	0.02	(0.01, 0.30)	<0.01
Hcy	2.49	11.63	(2.36, 54.37)	<0.01
TIR	-2.33	0.19	(0.02, 0.33)	0.01

**Table 4:** ROC curve analysis of DPN.

	AUC	SE	*P*	CI95%
TIR	0.86	0.04	<0.01	0.71, 0.92
Hcy	0.98	0.01	<0.01	0.00, 1.00
HDL-C	0.78	0.04	0.02	0.64, 0.89
HbA1c	0.82	0.06	<0.01	0.70, 0.93

## Data Availability

The datasets used and analyzed during the current study are available from the corresponding author upon reasonable request.
